# Evaluation of Ideological and Political Education under Deep Learning Neural Network

**DOI:** 10.1155/2022/9490017

**Published:** 2022-08-10

**Authors:** Binqiang Li, Huizhen Wang

**Affiliations:** ^1^College of Education, Zhejiang Normal University, Jinhua 321004, Zhejiang, China; ^2^College of Education, Xinzhou Normal University, Xinzhou 034000, Shanxi, China; ^3^College of Marxism, Xinzhou Normal University, Xinzhou 034000, Shanxi, China

## Abstract

Under the background of the rapid development of the new generation of information technology, artificial neural networks (ANNs) have made some progress in the evaluation research of various courses in colleges and universities. However, there is little research on the application of ANNs in Ideological and Political Education (IPE) courses. Based on this, this work attempts to introduce the Backpropagation Neural Network (BPNN) into the evaluation system of IPE courses. Firstly, the structure and characteristics of the BPNN are given, and it is optimized by the genetic algorithm based on its characteristics. Secondly, the theoretical framework of IPE course evaluation is established, and the corresponding evaluation model is constructed using the optimized BPNN. Finally, a questionnaire survey is designed to analyze the current situation of IPE evaluation in colleges and universities, and a simulation experiment is set up to test the BPNN evaluation model before and after optimization. The results are as follows. First, there are mainly five evaluation methods for IPE courses in Chinese colleges and universities: 6/4, 3/7, 2/2/6, 5/5, and 3/3/4. Second, the training error value of the BPNN model is in the interval (−2.3, 2.2), and when the number of cycles is 552, the error is infinitely close to zero. Thirdly, the training error value of the optimized BPNN model is in the interval (−0.22, 1.2), and when the number of cycles is 775, the error is infinitely close to zero. Fourthly, the error between the output value of the optimized BPNN model and the expert score value is generally smaller than the error value before optimization. This work aims to provide a theoretical reference for the further application of neural network technology in the evaluation of IPE.

## 1. Introduction

Education is a special practical activity. The practitioner is human, and the object of practice is human. The educational purpose of the ideological and political theory courses directly points to people's thoughts, which is very challenging. A scientific and effective evaluation mechanism plays an important role in promoting the education of ideological and political theory courses [1]. However, the current evaluation mechanism of Ideological and Political Education (IPE) still relies on the examination paper. It is undeniable that some schools have arranged social practice projects at the same time as the examination, which has improved the scientificity of the evaluation results of the ideological and political theory course and increased the students' social practice ability. However, the curriculum innovation has not brought about the synchronous innovation of the evaluation mechanism. As a branch of social science, ideological and political theory cannot rely on various instruments and equipment like the research and evaluation of natural science, nor can it be pushed back in failure. In the process of ideological and political theory research and teaching, scholars themselves are used as research tools for scientific research. However, with the development of modern science and technology, some available scientific and technological means do not seem to be used in the evaluation mechanism of ideological and political theory courses. The current evaluation mechanism of ideological and political theory courses is not coordinated with the development of modern science and technology [2]. At present, scholars in China have conducted research on the meaning of the teaching effectiveness of IPE. In these studies, it is believed that “the teaching effectiveness of IPE course is the actual effect of systematic Marxist theory and IPE for college students, helping college students establish a correct world outlook, outlook on life, and values and improving college students' ability to analyze and solve problems using Marxist positions, viewpoints, and methods.” This study finds that the definition of this connotation has a high degree of recognition in the academic circles and has been cited by many scholars [3]. The definition of the teaching effectiveness of IPE courses must be comprehensively considered [4]. In addition, the effectiveness of IPE to some extent depends on the words, deeds, and psychology of college students in the study of ideological and political theory courses. Some researchers have studied students' psychology and behavior to analyze the effectiveness of classroom teaching of ideological and political theory courses in colleges and universities [5].

Deep learning (DL) is a new technology in artificial intelligence. This concept was proposed by Professor Hinton, a British artificial intelligence expert, and others. It mainly refers to “using the multi-layer abstraction mechanism of the human brain to simulate the learning process of the human brain through the neural network to achieve the abstract expression of a large amount of data in the real world.” More importantly, the practice has proved that “DL can acquire the potential intrinsic features or rules of natural images, video, voice, music, and other data with potentially complex structural rules.” From this point of view, DL technology has a technical support function for the IPE theory course. In practice, the innovation of IPE evaluation can be explored according to the evaluation needs of ideological and political courses and the corresponding model of DL technology. Among them, the neural network technology in the DL technology is a key technology [6]. The development of the neural network is very tortuous. It originated from the pioneering work of neuron anatomist McCulloch and mathematical genius Pitts in 1943. They first proposed the McCulloch-Pitts model in the Journal of the Biophysical Society. The model theoretically demonstrated that as long as there were enough simple neurons connected and operating in synchrony, the network could complete the computation of any known function. In 1949, physiologists clearly stated the Hebb adjustment rule for neuron connection weights in the book. Its ideas provided a source of inspiration for the design of later learning systems and adaptive systems [7]. In 1957, the concept of perceptron was proposed, which gave a new method to solve problems such as pattern recognition [8]. Afterward, the doubts suffered by neural networks in the 1960s were resolved in the 1980s. Since then, neural networks had once again ushered in a period of prosperity. In 1982, a new form of calculation was described based on the idea of the energy function, which introduced a feedback network with symmetric synaptic connections into neural networks [9]. In 1983, the simulated annealing algorithm was reported [10]. The backpropagation algorithm was proposed in 1986 [11]. In 1988, the multilayer feedforward network designed based on the radial basis function came out [12]. Research on neural networks has flourished since then.

According to the analysis of the literature, there are still many areas to be strengthened in the reform of IPE in colleges and universities at this stage. Its educational model has not yet fully adapted to the needs of social and economic development, the teaching structure and system mechanism are not reasonable, and the teaching quality needs to be enhanced. This work will introduce neural network technology into the IPE evaluation system and set up experiments to verify its effect. This paper first introduces the relevant theory of the backpropagation (BP) neural algorithm, and the theoretical framework of the IPE course evaluation system is constructed. The Backpropagation Neural Network (BPNN) is introduced into it, and experiments are set up to verify the effectiveness of the constructed model. The innovation is that the genetic algorithm (GA) is used to optimize the BPNN, and the purpose of reducing the model error is achieved by adjusting the network weights. The purpose is to realize the evaluation system of IPE in colleges and universities to assist teachers' teaching and improve the quality of teaching.

## 2. Methods

### 2.1. Neural Network

#### 2.1.1. The Structure and Characteristics of the BPNN

The hidden layer of the BPNN can have one or more layers. The topology of the BPNN is shown in Figure 1 [13].

In Figure 1, *X*_*N*_ is the input value, and *Y*_*N*_ is the output value.

BPNN has three typical characteristics. First, it is composed of multiple layers. The neurons in the adjacent layers are fully connected, and the neurons in the same layer are not connected. Second, the network training process is carried out according to the error backpropagation algorithm. The signal flows from the input layer of the network through the hidden layer to the output layer. When the network weights are trained, the network weights are corrected from the output layer to the input layer in the direction of reducing the error. The process is repeated until the error tends to be extremely small. Third, the activation function of the network is differentiable, usually a Sigmoid function or a linear function [14]. The Sigmoid function is divided into the Log-Sigmoid function and Tan-Sigmoid function [15]. The expressions and strings of each function are as follows.

The linear function string is ‘purelin,' and the expression is

(1) $$\begin{array}{c} f\left(x\right)=x. \end{array}$$

The Log-Sigmoid function string is ‘logsig,' and the expression is

(2) $$\begin{array}{c} f\left(x\right)=\frac{1}{1+e^{-x}},\;\left(0<f\left(x\right)<1\right). \end{array}$$

The Tan-Sigmoid function string is ‘tansig,' and the expression is

(3) $$\begin{array}{c} f\left(x\right)=\frac{2}{1+e^{-x}}-1,\;\left(-1<f\left(x\right)<1\right). \end{array}$$

#### 2.1.2. The Training Process of the BPNN

The learning and training of the BPNN usually need to go through three stages. The first stage is the process of data preprocessing, which normalizes the collected sample data. The second stage is to build a reasonable network model and set the weights and thresholds of the network. The output of each neuron is calculated from the first layer of the network. The third stage is to reversely calculate the weights and thresholds from the network output layer in the direction of error reduction according to the training results and make improvements based on it [16]. These three stages alternate repeatedly until the network reaches its expectations. When a network algorithm is written, the number of network layers is determined based on the sample. Then, there is the training of the network. A complete BP network training process is revealed in Figure 2.

*(1) Normalization of Sample Data*. In practice, the size of network input data varies, so some values may be very large. This will lead to slow network convergence and a long training time. The input samples of the network are generally preprocessed before training to solve this problem. The normalization process of data is to map the input data into [0, 1], [−1, 1], or smaller regions [17]. In Matlab data processing, normalization can use premnmx, postmnmx, and tramnmx. The premnmx function is to normalize the two matrices of *p* and *t* to the [−1, 1] interval. The syntax is as follows:

(4) $$\begin{array}{c} \left[p\left(n\right),\min\left(p\right),\max\left(p\right),t\left(n\right),\min\left(t\right),\max\left(t\right)\right]=\text{premnmx}\left(p,t\right). \end{array}$$

In equation (4), *p*(*n*) and *t*(*n*) are the matrices generated by the row normalization of the *p* and *t* matrices, respectively. min(*p*) and min(*t*) are the minimum values of each row of the *p* and *t* matrices, respectively. max(*p*) and max(*t*) are the maximum values of each row of the *p* and *t* matrices, respectively.

*(2) Creation of the Network*. A basic form of the feedforward network creation function, newff function, is as follows:

(5) $$\begin{array}{c} \text{netnewff}\left(A,B,\left\{C\right\},{\;}^{\prime \prime }\text{train Fun}{\;}^{\prime \prime },{\;}^{\prime \prime }\text{BLF}{\;}^{\prime \prime },{\;}^{\prime \prime }\text{PF}{\;}^{\prime \prime }\right). \end{array}$$

In equation (5), *A* represents an *n* × 2 matrix. *B* represents a *k*-dimensional vector whose elements are the number of nodes in the hidden layer of the network. *C* represents a *k*-dimensional string row vector, where each component represents the activation function of the corresponding layer of the network. Train Fun is the training algorithm selected for learning. BLF represents the weight of the BP network. PF is the performance function, which defaults to ‘mse' [18].

*(3) Reasonable Configuration of Network Parameters*. The commonly used network configuration parameters are generally adopted here.

*(4) Training of the Network*. The syntax of the network training train function is

(6) $$\begin{array}{c} \left[\text{net},\text{tr},Y1,E\right]=\text{train}\left(\text{net},X,Y\right). \end{array}$$

In equation (6), *X* and *Y* are the actual input and target output of the network, respectively. tr is the training tracking information. *Y*1 represents the actual output of the network. *E* is the error matrix of the network.

#### 2.1.3. BP Algorithm with Variable Learning Rate

In the standard BP algorithm, the learning rate is a fixed parameter, which will not change with the training during the learning and training process. The learning rate greatly impacts the network. A learning rate that is too small will slow down the convergence speed of the network and prolong the training time. An excessive learning rate will cause network oscillation and instability [19]. At different stages of learning and training, the learning rate required by the network may not be a fixed value, so it is unrealistic to determine the appropriate learning rate before training. If the value of the learning rate can be adjusted adaptively according to the actual training situation, it will greatly improve the stability of the network [20].

The BP algorithm with a variable learning rate can automatically correct the learning rate according to the change of the error performance surface. The adaptive process of the learning rate is achieved by multiplying by an increment or decrement factor.

(7) $$\begin{array}{c} \eta \left(k+1\right)=\left\{\begin{array}{c} K_{\text{inc}}\eta \left(k\right)E\left(k+1\right)<E\left(k\right)\\ K_{\text{dec}}\eta \left(k\right)E\left(k+1\right)>E\left(k\right) \end{array}.\right. \end{array}$$

If the error approaches the target in a smaller form, it indicates that the correction direction is right at this time, and the step size should be added. Multiplying the learning rate by an increment factor *K*_inc_ can promote the learning rate of the network. If the difference between the error and the set target exceeds a certain range, it indicates that the correction is excessive at this time, and the step size should be reduced. The learning rate is multiplied by the decrement factor *K*_dec_ to reduce the learning rate while undoing the previous correction process [21].

The variable learning rate BP algorithm can greatly improve the performance, convergence speed, and stability of the neural network. Therefore, this work applies the variable learning rate momentum BP algorithm to the evaluation of IPE courses, and the training function is ‘traindx.'

### 2.2. Genetic Algorithm

#### 2.2.1. Principle of GA

GA is a computational model that seeks optimal solutions by imitating biological evolution and natural selection processes [22]. GA starts with a population that represents a set of solutions to a problem, which is a combination of genetically encoded individuals. The chromosomes carried by each individual are used as the carrier of genetic material to determine the basic characteristics of each individual. Since the genetic coding work is very cumbersome, people usually simplify it. After the original population is generated, it evolves from generation to generation according to the principle of “survival of the fittest.” The population formed by the evolutionary excellent individuals will be more suitable for the living environment than the original population through the selection, crossover, and mutation operations of each generation of individuals [23]. The result obtained after decoding by the optimal individual in the last generation population can be regarded as the global optimal solution for training.  Figure 3 shows the flow of GA.

#### 2.2.2. Basic Operation of GA

*(1) Chromosome Coding*. Coding chromosomes is the primary task of GA, and the quality of the coding process directly impacts the training results. Commonly used chromosome encoding methods include binary encoding, character encoding, and floating-point number encoding. The specific encoding method to be used needs to be determined through the analysis of actual problems [24].

*(2) Population Initialization*. Before genetic manipulation starts, it is necessary to generate an original population to participate in the subsequent evolutionary process. A population is composed of many chromosomes, and each chromosome has an initial solution. For now, there is no precise theory to guide population size. If the population size is too small, the network will converge quickly, but it may not be able to find the optimal solution. If the population size is too large, the network will converge slowly, and the training time will be too long. Therefore, the population size needs to be determined according to actual problems and reference experience settings, and the population can also be generated by random generation [25].

*(3) Fitness Function Design*. Whether an individual can be selected depends on the size of fitness. In general, the higher the individual fitness value, the greater the probability of survival. Individuals with low fitness tend to be eliminated in evolution. The fitness function is an independent individual. Its domain and functional form have fixed restrictions, and how to obtain its value needs to be set according to the actual problem [26].

*(4) Genetic Manipulation*. The genetic operation usually refers to three operation methods of selection, crossover, and mutation, which constitute the core content of GA. The survival of the fittest in the population is completed through the selection, crossover, and mutation of the population, and the evolution process of the entire population is completed [27].

### 2.3. The Theoretical Frame Design of IPE Courses Evaluation System

#### 2.3.1. Evaluation Function Design

The functions of the IPE course evaluation system are shown in Figure 4.

#### 2.3.2. Design of Evaluation Types

The evaluation of IPE courses has a wide range and many contents. The evaluation of IPE courses can be classified from different angles. The IPE course evaluation can be divided into the formative evaluation and summative evaluation from the perspective of the role and function of the IPE course evaluation [28].

### 2.4. Model Design of IPE Course Evaluation

#### 2.4.1. Design Principles of Evaluation Indicators

An indicator is a summary and definition of certain characteristics of activity. These characteristics can be measured and can reflect the nature and development law of the activity. The activities are promoted to the expected standards, specifications, and directions through the learning of features [29]. A system refers to a collection of things that are unified by interaction and dependence due to a certain connection. To sum up, the evaluation indicator system is an organic whole with an internal structure composed of a series of interrelated and mutually restrictive evaluation indicators [30]. In the IPE course evaluation activities, the most important point is to indicate the evaluation system. The indicator helps to concretize some general and ambiguous contents in evaluation activities. These contents are refined to each clear point to enhance the operability of the evaluation activities. The system should be constructed by the principles of systematicness, pertinence, practicality, and independence to reasonably and effectively construct an indicator system that truly reflects the intrinsic performance of the object being evaluated [31].

#### 2.4.2. Construction of Evaluation System

The evaluation of IPE courses should enrich the types and timing of evaluation and focus on the combination of process and results. The evaluation should also strengthen the supervision mechanism for students and advocate the use of various test modes. Students are evaluated at different periods to urge them to develop good study habits and interest in learning. This work analyzes the problems existing in the evaluation of IPE courses in vocational education, the principles of indicator design, and the existing theories. The refined IPE evaluation indicator system is demonstrated in Table 1.

#### 2.4.3. Construction of Evaluation Model of IPE Course Based on Optimized BPNN

The GA is used to optimize the weights of the BPNN to speed up the network convergence time and avoid the network from falling into the local optimum. The optimized BPNN model is displayed in Figure 5.

The evaluation model of the IPE course is obtained by combining the optimized BPNN with the content of the indicator system of the IPE course, as shown in Figure 6.

### 2.5. Experiment Design

#### 2.5.1. Questionnaire Design

This work adopts a combination of online questionnaire star and offline work distribution to study the composition of IPE course evaluation in colleges and universities at this stage. Besides, 150 questionnaires were distributed to 16 different institutions in China. The number of universities in the south is 8, accounting for 50%, and the number of universities in the north is 8, accounting for 50%.

#### 2.5.2. Simulation Experiment Design

This work summarizes the 20 groups of sample data obtained by summarizing the IPE course results of students in a higher vocational college. The simulation design is performed through the Matlab platform to verify the IPE evaluation model based on the BPNN and the effect of the BPNN model optimized by GA. Expert scoring is the result of each sample of data calculated according to the proportion of the indicator system. The first 15 sets of data are used as learning data for training the learning network model. The last five sets of data are test samples, which are used to compare the training errors to judge the performance of the obtained network model.

The training method of the sample data is to use the newff function to create a BPNN with 14 inputs and 1 output, and the number of hidden layer nodes is 8.

  Net = newff (minmax(pn), [1, 8, 14], {‘tansig', ‘tansig', ‘purelin'}, ‘traingdx');
  The network parameters are set reasonably.
  net.train Param.show = 5000; % shows the period of intermediate results.
  net.train Param.lr = 0.01; % learning rate.
  net.train Param.mc = 0.9; % momentum factor
  net.train Param.epochs = 3000; % maximum number of training sessions
  net.train Param.goal = 1*e* − 9; % the target accuracy to be achieved by training.

## 3. Results and Analysis

### 3.1. Current Situation of IPE Course Evaluation

The distribution results of the IPE course evaluation composition of different colleges and universities are obtained after a questionnaire survey is conducted on each school.  Figure 7 shows the results.

Figure 7 indicates that there are five main ways of evaluating IPE courses in Chinese colleges and universities. The first is the examination mode (6/4) consisting of the usual grades and final examinations, accounting for 60% and 40%, respectively. The second is the examination mode (3/7) consisting of the usual grades and final examinations, accounting for 30% and 70%, respectively. The third is the examination mode (2/2/6) consisting of usual grades, practical operations, and final examinations, accounting for 20%, 20%, and 60%, respectively. The fourth is the examination mode (5/5) consisting of the usual grades and the final examination, accounting for 50% and 50%, respectively. The fifth is the examination mode (3/3/4) consisting of usual grades, practical operations, and final examinations, accounting for 30%, 30%, and 40%, respectively. The above data shows that the composition of the IPE course examination mode of the 16 colleges and universities surveyed is diversified.

### 3.2. Evaluation Model Test Based on BPNN

#### 3.2.1. Training Results of Evaluation Model Based on BPNN

The Matlab platform is used to train the evaluation model of IPE courses based on the BPNN, and the results are shown in Figure 8.

Figure 8 reveals that the training error of the first 15 groups of data remains zero and does not change after the sample data is imported into the BPNN model for training. The training error of the last five groups of data fluctuates significantly, and the error value is in the interval (−2.3, 2.2). In addition, The mean square error of BPNN training decreases with the increase of the number of network loops. When the number of loops is 552, the mean square error of the network is infinitely close to zero. This shows that the BPNN has accuracy and good convergence, but there are still problems such as large errors and instability, so further optimization is needed.

#### 3.2.2. Comparison of Expert Scores and Model Prediction Results

The scores of the experts on the test samples and the prediction results of the model based on the optimized BPNN are shown in Table 2 and Figure 9. Figure 9 is a graphical representation of the data in Table 2.

From Figure 9, for the test sample data, the expert scores are 86, 82, 79, 90, and 86, respectively. The predicted values of the BPNN model are 86.2, 80.9, 76.8, 92.3, and 86.1, respectively. The error values are −0.2, 1.1, 2.2, −2.3, and −0.1, respectively. The above data show that the output value error of the BPNN model varies widely and is unstable.

### 3.3. Evaluation Model Test Based on Optimized BPNN

#### 3.3.1. Training Results of Evaluation Model Based on Optimized BPNN

The Matlab platform is adopted to train the optimized BPNN after the GA is used to optimize the BPNN. The results are shown in Figure 10.

From Figure 10, the training error of the first 15 groups of data remains zero after the sample data is imported into the optimized BPNN model for training. The training error of the last five groups of data fluctuates significantly, and the error value is in the interval (−0.22, 1.2). Furthermore, the mean square error of the optimized BPNN training decreases with the increase of the number of network loops. When the number of loops is 775, the mean squared error of the network is infinitely close to zero. This shows that the optimized BPNN has been significantly improved in both accuracy and convergence. Meanwhile, it also indicates that the IPE course evaluation model based on this model is practical.

#### 3.3.2. Comparison of Expert Scores and Model Prediction Results

Figure 11 shows the comparison between the expert's scores on the test samples and the prediction results of the model based on the optimized BPNN.

From Figure 11, for the test sample data, the expert scoring results are 86, 82, 79, 90, and 86, respectively, while the predicted values of the optimized BPNN model are 84.8, 80.8, 79.2, 90.1, and 86.2, respectively. The error values are −1.2, 1.2, −0.2, −0.1, and −0.2, respectively. The above data show that the error range of the output value of the BPNN model optimized by the GA is significantly reduced.

## 4. Discussion

IPE is one of the important measures to cultivate Chinese skilled talents. In recent years, the school-running system, school-running quality, and school-running model have been continuously innovated, upgraded, and improved under the promotion of the central and local governments. The scale of enrolment and the employment rate of graduates have increased significantly. IPE has entered the “fast lane” of development. The evaluation of IPE is the main means to reflect the development of the ideological and political courses of college students. The fairness and reasonableness of the evaluation results are directly related to whether students can correctly understand themselves, establish self-confidence, and improve themselves. As described in the literature on IPE, on the one hand, the connotation of IPE is significant. IPE is an important method to improve a person's ideological height, so it is worthy of a country's attention. On the other hand, the purpose of implementing IPE by the state is to directly help people's thoughts. Therefore, people can be firm in their hearts, have beliefs, and realize their values. This process is extremely challenging, which shows that a scientific and effective evaluation mechanism has a nonnegligible boosting effect on the educational work of ideological and political theory courses. Based on the above content, this paper further studies the evaluation model of IPE based on studying the evaluation model of Chinese IPE. In addition, the neural network technology in DL is integrated to build a scientific evaluation model. The model plays a very good role in both accuracy and prediction effect. The novelty is to optimize the constructed IPE evaluation model using GA. The prediction effect of the model has improved in both accuracy and speed. Furthermore, the model can also minimize the impact of human factors on evaluation activities, which is crucial to the development of students' IPE curricula.

## 5. Conclusion

This work establishes a suitable evaluation system for IPE courses based on the current situation of vocational education development and the investigation of the composition ratio of evaluation. The neural network optimized by GA is introduced to quantify complex indicators. The neural network learning model is constructed through the Matlab platform. The rationalized results are acquired through training, adjustment of weights and parameters, and optimization of GA. The results show that the evaluation methods of IPE courses in Chinese colleges and universities are diversified and not uniform. The evaluation model of IPE courses based on the BPNN has accuracy and good convergence, but there are still problems such as large errors and instability. The IPE course evaluation model optimized by GA has been improved obviously in accuracy and convergence. In addition, the error range of the output value of the BPNN model optimized by the GA is significantly reduced. The inadequacy is that only a small number of colleges and universities in China have been surveyed, and there may be other IPE course evaluation systems that have not been discovered. In the follow-up, the scope of the questionnaire will continue to be expanded to obtain a complete evaluation system for IPE courses. This work aims to explore a scientific evaluation system of IPE courses to reduce the impact of human factors on evaluation activities.

## Figures and Tables

**Figure 1:** BPNN topology diagram.

**Figure 2:** BPNN training process.

**Figure 3:** GA flowchart.

**Figure 4:** Functions of the IPE course evaluation system.

**Figure 5:** Optimization process of BPNN model based on GA.

**Figure 6:** The neural network model for IPE course evaluation.

**Figure 7:** Composition of IPE courses in different colleges and universities.

**Figure 8:** Training results of the IPE course evaluation model based on the BPNN. (a) The variation graph of the training error of the model. (b) The variation graph of the mean square error of the model.

**Figure 9:** Comparison of expert scores and model predictions.

**Figure 10:** Training results of the IPE course evaluation model based on the optimized BPNN. (a) The change graph of the training error of the improved model. (b) The change graph of the mean square error of the improved model.

**Figure 11:** Comparison of the expert scoring and the prediction results of the optimized model.

**Table 1:** IPE course evaluation indicator system.

First-level indicator	Secondary indicators	Score
Classroom situation (35%)	Punching in class	20
	Classroom style	20
	Classroom tasks	40
	Interaction in class	20

Extracurricular extension (20%)	Extracurricular reading	70
	Knowledge competition	30

Aptitude test (45%)	In-class test	20
	Exam performance	20
	Final grade	60

**Table 2:** Comparison of expert scoring results and model prediction results.

Test sample serial number	1	2	3	4	5
Expert scoring results	86	82	79	90	86
Model predictions	86.2	80.9	76.8	92.3	86.1
Error	−0.2	1.1	2.2	−2.3	−0.1

## Data Availability

The data used to support the findings of this study are available from the corresponding author upon request.
